# Isoliquiritigenin Suppressed Esophageal Squamous Carcinoma Growth by Blocking EGFR Activation and Inducing Cell Cycle Arrest

**DOI:** 10.1155/2020/9259852

**Published:** 2020-03-08

**Authors:** Liping Ye, Junjie Zhang, Yu Zhang, Binbin Gu, Hongyuan Zhu, Xinli Mao

**Affiliations:** ^1^Department of Gastroenterology, Affiliated Tai Zhou Hospital of Wenzhou Medical University, No.150 Ximen Road, Linhai City, Taizhou 317000, China; ^2^Department of Gastroenterology, Tongji Hospital, Tongji University School of Medicine, Shanghai 200065, China

## Abstract

Isoliquiritigenin (ILQ) is a natural product isolated from licorice root which has served as traditional Chinese medicine for a long time. Recently, the antitumor effects of ILQ have been widely studied in various cancers, but the role and related mechanisms of ILQ in esophageal squamous carcinoma cells (ESCC) are still poorly understood. In our studies, ILQ showed profound antitumor activities in ESCC cells. In vitro, ILQ substantially inhibited cell proliferation and anchorage-independent growth in a panel of human ESCC cells. Mechanism studies showed that EGFR signaling pathway played an important role for ILQ to exert its antitumor activity in ESCC. Exposure to isoliquiritigenin substantially decreased EGF-induced EGFR activation and its downstream Akt and ERK1/2 signaling pathway. EGFR knockdown with shRNA in ESCC cell significantly reduced the sensitivity of cancer cells to ILQ. Moreover, it was found that ILQ had a significantly inhibitory effect on AP-1 family, the protein of Jun and Fos subfamilies was substantially downregulated, and the transcriptional activity of AP-1 family was dramatically suppressed by ILQ. By reducing the expression of cyclin D1, ESCC cells were induced G0/G1 arrest, and cell division was substantially blocked. Finally, the antitumor potency of ILQ was validated in xenograft models and the tumor growth was prominently restrained by ILQ. Briefly, our study showed that ILQ, or its analogue, appeared to be a promising new therapeutic agent for ESCC management.

## 1. Introduction

Esophageal carcinoma is a malignancy with high mortality worldwide and caused about 500,000 deaths per year [1]. In China, the number of new cases and deaths each year is 286,700 and 211,000, ranking sixth and fourth, respectively [2]. Unlike most esophageal cancers in western countries, which are adenocarcinoma (EA), more than 85% of esophageal cancers in China are squamous cell carcinoma (ESCC). The high incidence of ESCC is considered to be associated with alcohol and tobacco consumption [3]. In terms of the biological and genetic background, EA shares some similarities with gastric cancer, while ESCC possesses more common genetic characteristics with head and neck squamous cell carcinoma. Large-scale sequencing of ESCC revealed that the abnormalities of multiple pathways including tyrosine kinase receptors, cell cycle regulation, and chromosome restructuring contributed to the development of ESCC [4, 5].

The epithelial growth factor receptor (EGFR), which belongs to the receptor tyrosine kinase family, has a crucial role in tumor development. Physiologically, the activation of EGFR is induced by its ligand, which caused its dimerization and phosphorylation. Then the downstream MAP kinase pathway and phosphatidylinositol 3-kinase (PI3K)/Akt pathway was activated and initiated a series of cellular processes such as cell proliferation, migration, and metabolism. Owing to its importance, in some tumor types such as lung adenocarcinoma, the somatic mutations of EGFR can act as a driver to accelerate tumor growth. And the tumors with EGFR mutations have shown great response to EGFR inhibitors [6]. Although the sensitive mutations were rare in ESCC, EGFR overexpression was frequently observed and found to be closely related to clinical stages, tumor invasion, and patient survival [7]. Some studies also reported the overexpression of EGFR was significantly correlated with the lymph node metastasis [8]. In addition to overexpression, gene amplification of EGFR was also identified in ESCC tissue. The analysis of survival demonstrated that the patients with low copy number had longer survival in contrast with those of high EGFR amplification [9, 10].

Licorice is a plant widely cultivated in China, and its root is used as traditional herb for the therapy of different diseases [11]. The extracts from its root are used as food additives in candies, soft drinks, and toothpaste as well [12]. Recently, the pharmacology studies showed that the licorice extracts had antioxidative, anti-inflammation, and other biological functions [13, 14]. Isoliquiritigenin (ILQ) is a chalconoid isolated from licorice root extract. In addition to the same pharmacological effect as licorice, ILQ also exerted antidiabetic and antispasmodic activities [15, 16]. Recently, multiple studies had investigated the effect of ILQ on cancers, and ILQ has exhibited profound antitumor abilities against breast cancer, hepatocellular carcinoma, colon cancer, cervical cancer, prostate cancer, endometrial cancer, and so on [17–22]. So far, the direct target of ILQ in tumor cells has not been elaborated, but several nonspecific mechanisms modulated by ILQ have been reported. ILQ was reported to decrease the expression of matrix metallopeptidases (MMPs) and reduce cancer cell migration [23]. Through mediation of cell death program and the suppression of extracellular matrix, ILQ showed substantial potency in uterine leiomyoma [24]. Besides that, induction of cell apoptosis by ILQ has been extensively investigated. Different mechanisms including activation of ataxia telangiectasia-mutated (ATM), upregulation of p53 and p21, and G2/M phase arrest, the changes of proteins in apoptosis family were suggested to correspond with apoptosis induction by ILQ [21, 25, 26].

In the present study, we mainly evaluated the antitumor abilities of ILQ in esophageal squamous cell carcinoma in vitro and in vivo. Further, we illustrated the potential target and related mechanisms of action of ILQ. This study provided some insights into the biological functions of ILQ or related analogues in the prevention and treatment of esophageal squamous cell carcinoma.

## 2. Material and Methods

### 2.1. Cell Lines and Reagents

The esophageal squamous cell carcinoma (ESCC) cells KYSE140, KYSE520, and TE1 were obtained from the Cell Bank of the Chinese Academy of Sciences (Shanghai, China). All cells were subjected to mycoplasma examination and cytogenetically test and cultured with completed culture medium (basic medium supplemented with 10% fetal bovine serum) according to the standard protocols. The compound isoliquiritigenin was purchased from Selleck Chemicals (Houston, TX). Recombinant human EGF was product of R&D. The primary antibodies used in this study including anti-p-EGFR (Tyr1068) (#3777), anti-EGFR (#4267), anti-p-Akt (S473) (#4060), anti-Akt (#4691), anti-p-ERK1/2 (Thr202/Tyr204) (#4370), anti-ERK1/2(#4695), anti-c-Jun (#9165), anti-JunB (#3746), anti-JunD (#5000), anti-FosB(#4691), anti-c-Fos (#2251), anti-Fra1(#5281), anti-Cyclin D1(#55506), anti-*β*-actin (#3700), and anti-Histone H3 Ser10 (#53348) were products of Cell Signaling Technology (Danvers, MA). Lentivirus plasmids (pLKO.1-shEGFR) were purchased from Thermo Scientific (Huntsville, AL, USA).

### 2.2. Cell Proliferation Assay

Briefly, 100 *μ*l ESCC cell suspension was plated into a 96-well plate with the density of 3,000 cells/well and then incubated with indicated concentrations of ILQ (final concentration is *μ*M, respectively). After the treatment of different times, cell viabilities were determined with the CellTiter 96 Aqueous One Solution Cell Proliferation Assay (Promega) by following the standard protocol provided by the manufacturer.

### 2.3. Soft Agar Assay

The soft agar assay was performed as described previously [27]. Briefly, 3 ml basal medium Eagle's medium containing 0.6% agar, 10% FBS, and various concentrations of ILQ was loaded into a 6-well plate. After the agar was solidified, ESCC cells were digested and harvested by centrifugation, and then the cell pellets were resuspended with the culture medium containing 10% FBS and 0.3% agarose, and cell density was adjusted to 8,000 cells/ml. 1 ml cell suspension was seeded on the top of solidified agars and then treated with different concentrations of ILQ. The cells were maintained in the incubator for 2 weeks. The number of cell colonies in the agar was observed and counted using the microscope.

### 2.4. Cell Cycle Analysis

KYSE140 cells were seeded into 6-well plate and maintained overnight, and then cells were treated with various concentrations of ILQ for 24 h. After that, the cells were harvested and fixed with precold 70% ethanol at 4°C for at least 24 h. After washing, the cells were incubated with 50 *μ*g/ml ribonuclease A at 37°C for 30 min and then stained with 50 *μ*g/ml propidium iodide at room temperature for 15 min avoiding light. The cell cycle was analyzed by FACSort Flow Cytometer (BD, San Jose, CA, USA).

### 2.5. AP-1 Luciferase Reporter Assay

The Dual-Luciferase reporter assay was performed as described previously [28]. Briefly, the ESCC cells were seeded in a 24-well plate and transfected with pGL3-AP-1 (#40342, Addgene) or pGL3-Basic control vector along with the renilla luciferase reporter construct pRL-SV40for 24 h. Cells were then treated with isoliquiritigenin for another 24 h and harvested for firefly luciferase and renilla luciferase activity determination using the Dual-Luciferase reporter assay system (#E1910; Promega, Madison, WI, USA). Renilla luciferase activity was used as a control for transfection efficiency.

### 2.6. Western Blotting

After the treatment of ILQ, the cells were harvested and lysed with NP40 lysis buffer (50 mmol/L Tris-HCl, pH 8.0; 150 mmol/L NaCl; 0.5% NP40) supplemented with protease cocktail on ice (Roche, Germany). The proteins in cell lysates were extracted by high-speed centrifugation (12000g) at 4°C for 10 min, the supernatant was collected, and protein concentration was determined using the BCA protein assay kit (Thermo Fisher Scientific, Waltham, MA). The protein sample (20 *μ*g/lane) was mixed with loading buffer and subjected to SDS-PAGE electrophoresis and then electrically transferred to nitrocellulose membrane. The membrane was then blocked using 5% nonfat dry milk in PBS and incubated with primary antibody overnight at cold room. After washing with PBST, the membrane was incubated with HRP-labeled second antibody. The probed proteins were visualized at the darkroom using the ECL chemiluminescence reagents (Thermo Fisher Scientific, Waltham, MA).

### 2.7. Immunofluorescence Assay

KYSE-140 cells were seeded into 24-well plate preloaded with a coverslip and treated with different concentrations of ILQ for 24 h. After washing with PBS for 3 times, the cells were fixed with cooled 4% paraformaldehyde on ice for 2 h and then incubated with 0.25% Triton X-100 for 10 min on ice. After incubation with blocking solution (5% BSA in PBS solution), the coverslip was washed with PBS solution for 5 min and then incubated with primary antibody in a humid chamber at 4°C overnight. The specimen on the slides were washed with PBS and hybridized with FITC-labeled secondary antibody at room temperature for 1 h. Then the coverslip was counterstained with propidium iodide (PI), mounted, and observed with fluorescence microscope.

### 2.8. Lentiviral Infection

To generate lentiviral particles, the plasmid pLKO.1-sh-EGFR, psPAX2 (#12260, Addgene), or pMD2.G (#12259, Addgene) was cotransfected into HEK-293T cells with PSPAX2 and PMD2.G. The transfected 293T cells were maintained at the incubator for 48 h, and viral supernatant fraction was collected and filtered through a 0.45 *μ*m filter. For knockdown stable cell generation, the cells were cocultured with the viral supernatant together with 6 *μ*g/mL polybrene overnight. Stable cells were selected by 2 *μ*g/mL puromycin for 3 days.

### 2.9. Tumor Xenograft Experiment

This study was approved by Animal Care and Use Committee of Wenzhou Medical University and all operations strictly follow the Guide for the Care and Use of Laboratory Animals. Six-eight weeks old female Balb/c athymic nude mice were used in animal studies. Briefly, KYSE140 cells were subcutaneously injected into the right flank of mice at a concentration of 2 × 10^6^ cells/mice. When the tumor volume reached about 100 mm^3^, mice with appropriate tumor size were selected and randomly assigned to vehicle or treatment group. ILQ (10 mg/kg) or vehicle control was administrated every two days by intraperitoneal injection. Body weight was monitored, and tumor volume was measured twice a week with caliper and determined as (length × width^2^)/2.

### 2.10. Immunohistochemical (IHC) Staining

IHC staining was performed as described previously [29]. Briefly, xenograft tumors were embedded in parafﬁn and then cut into tissue slide sections. The slides were deparaffinized, hydrated, and immersed into 3% H_2_O_2_ for 10 min for eliminating endogenous peroxidase activity, followed by antigen retrieval using a microwave oven. Tissues were blocked with 5% goat serum at room temperature for 1 h and incubated with primary antibody at 4°C overnight. After incubation with the second antibody, the target protein was visualized with 3,3-diaminobenzidine (DAB) substrate. Hematoxylin was used for counterstaining.

### 2.11. Statistical Analysis

The statistical analysis was performed using SPSS software (version 16.0). Quantitative data were expressed as mean values ± standard deviation, and the significant differences were assessed by a two-tailed Student's *t*-test or one-way ANOVA. *p* < 0.05 was considered to be statistically significant.

## 3. Results

### 3.1. Isoliquiritigenin (ILQ) Inhibited ESCC Proliferation In Vitro

Firstly, the potency of ILQ against esophageal squamous carcinoma cells was determined by MTS assays. As shown in Figures 1(b)–1(d), in three tested ESCC cells KYSE-140, KYSE-520, and TE-1, ILQ had demonstrated profound antitumor activity, and the cell viability was significantly decreased in a dose- and time-dependent manner. Moreover, the ESCC cells were incubated with different concentrations of ILQ, and colony formation in soft agar was examined. In contrast with the control group in which a number of cell clones were observed, with the increase of ILQ, the number of clones formed in the agars was dramatically decreased; at the high concentration of 20 *μ*M, the number of cell colonies dropped more than 80% (Figures 1(e)–1(g)).

### 3.2. Isoliquiritigenin (ILQ) Inhibited EGFR Activation in ESCC Cells

EGFR is a crucial signaling pathway, and frequently with overexpression in most ESCC cells, the effect of ILQ on EGFR activation was examined. As shown in Figure 2(a), after incubation with ILQ, the phosphorylation of EGFR was dose-dependently decreased, indicating the activity of EGFR was suppressed. Moreover, with EGFR inhibition, the phosphorylation of ERK and AKT, two major downstream signaling molecules, were both significantly reduced. To clarify the specificity of EGFR inhibition, we determined the effect of ILQ on EGF-induced EGFR activation. After starvation, the phosphorylation of EGFR in ESCC cells was very low, and EGF substantially stimulated the activation of EGFR, but EGF-induced phosphorylation of EGFR was substantially suppressed by ILQ in a dose- and time-dependent manner (Figures 2(b) and 2(c)), suggesting that ILQ inhibited EGFR in a direct way. Furthermore, we also investigated the role of EGFR played in ILQ-mediated antitumor activities. EGFR knockdown cells were generated with specific shRNAs, and the activity of ILQ was studied. As shown in Figures 2(e) and 2(f), in parent cells, cell clones formed were significantly decreased after ILQ treatment. After transfection with EGFR-shRNA, the ability of colony formation had been affected in contrast with GFP-shRNA. However, the sensitivity of EGFR deficient cells to ILQ was substantially decreased, suggesting that the inhibition of EGFR signaling pathway played an important role for ILQ to exert its antitumor ability.

### 3.3. Isoliquiritigenin (ILQ) Suppressed the Transcriptional Activity of AP-1

AP-1 is an important transcription factor that regulates a series of cellular biological functions, such as cell proliferation, survival, and transformation. We have investigated the effect of ILQ on AP-1 activities. In ILQ-treated ESCC cells, the expression of JunB and JunD, which belong to the Jun subfamily, was significantly decreased. Meanwhile, other proteins in the Fos subfamily, including FosB, c-Fos, and Fra1, were also substantially decreased after ILQ treatment (Figures 3(a) and 3(b)). To confirm the effects of ILQ on AP-1 transcriptional activities, AP-1 luciferase reporter assay was used to evaluate the transcriptional activity. As shown in Figures 3(c) and 3(d), after the treatment of ILQ, the activities of luciferase were dose-dependently decreased, suggesting the transcriptional activity of AP-1 was substantially inhibited after exposure to ILQ. Since the downstream signaling pathway of EGFR, such as MAPK, is involved in the regulation of AP-1 transcriptional activity, we also investigated the role of EGFR inhibition in ILQ-mediated AP-1 suppression. In EGFR knockdown cells, ILQ-induced suppression of AP-1 was significantly attenuated (Figure 3(e)), implying the inactivation of EGFR by ILQ at least partially contributed to the inhibition of AP-1.

### 3.4. ILQ-Induced Cell Cycle Arrest by Reducing Cyclin D1

Phosphorylation of histone H3 (p-H3) is an important biomarker of cell mitosis, and its expression is closely associated with cell proliferation. The result of immunofluorescence showed that after exposure to ILQ, the intensity of p-H3 was dose-dependently decreased, suggesting the cell division was blocked (Figure 4(a)). Next, we analyzed the cell phase distribution in ILQ-treated cells, as shown in Figure 4(b), after the treatment of ILQ, the proportion of cells in the G0/G1 phase increased in a dose-dependent manner, suggesting ILQ could cause cell cycle arrest. Furthermore, we examined the effect of ILQ on proteins involved in the mediation of G0/G1 phase progression. In Figure 4(c), the results showed that ILQ dose-dependently inhibited the expression of cyclin D1, while no visible change of CDK4 and CDK6 was observed.

### 3.5. ILQ Inhibited Xenograft Growth In Vivo

Finally, the activity of ILQ against ESCC was studied in the KYSE-140 xenograft model. As the results shown in Figure 5(a)–5(c), ILQ at the dose of 10 mg/kg had demonstrated profound antitumor potency. Compared with the tumor volume at the dosing begins, the tumor growth in vehicle group was rapid, and the average volume reached 400 mm^3^. However, after ILQ treatment, the tumor growth was suppressed and no obvious growth was observed in contrast with the volume at the beginning. During the treatment, the body weight of mice had no significant change, indicating that ILQ was safe at this pharmacodynamic dose and tolerable in mice (Figure 5(d)). Furthermore, the result of immunohistochemistry staining showed that, in ILQ-treated tumor tissue, the phosphorylation of EGFR was significantly reduced. Meanwhile, the intensity of Ki67, a well-known biomarker of tumor cell proliferation, was also dramatically decreased (Figure 5(e)).

## 4. Discussion

With the development of diagnosis and treatment, the overall survival of cancer patients has improved significantly in the recent years. In contrast, because of the high heterogeneity, the five-year survival rate of esophageal squamous cell carcinoma, especially that in advanced stage or with node metastasis, is relatively low, only 15–25% [30]. Compared with traditional radiochemotherapy, the cancer immunotherapies represented by PD-1/PD-L1 antibodies have brought new hopes. However, owing to the low response rate and the lack of definite biomarkers of immunotherapy, new treatment strategies are still in urgent need. It is a critical approach to discover useful components from traditional Chinese medicines with long history of clinical applications. In our studies, we demonstrated that isoliquiritigenin (ILQ), a chalconoid derived from the root of liquorice, exhibited substantial antitumor potency against ESCC through inactivation of EGFR signaling pathway. With the suppression of EGFR, the activities of downstream ERK and AKT were inhibited and the transcriptional activity of AP-1 was reduced, which gave rise to the decrease of cylcinD1 expression and cell cycle G0/G1 arrest (Figure 6).

As reported by the previous study [22], ILQ at the concentration of 20 *μ*M had no toxicity on normal cells. Therefore, we used 20 *μ*M as the top concentration to evaluate the antitumor potency in ESCC cells; in vitro, ILQ inhibited ESCC cell proliferation and colony formation in a dose-dependent manner, suggesting that ILQ suppressed ESCC cells in a specific way. Due to the hepatic and intestinal metabolism, the bioavailability of oral administration of ILQ is relatively low. Therefore, in animal study, ILQ was dosed by intraperitoneal injection, and the tumor growth was suppressed at the dose of 10 mg/kg.

It is consolidated that the dysregulation of EGFR activity is closely associated with tumor development. The success of the first to the third generation of EGFR inhibitors such as gefitinib, afatinib, and osimertinib in non-small cell lung cancer proved that targeting EGFR pathway in cancer cells is an effective method [31–33]. Although no obvious somatic mutation of EGFR was detected in esophageal squamous cell carcinoma, EGFR amplification or overexpression was frequently observed, which suggested that inhibition of EGFR activity was a strategy with great potentials. The preliminary results of EGFR inhibitors in clinical trials also confirmed this hypothesis. Icotinib, an EGFR inhibitor, under the patients' selection with EGFR overexpression or amplification, has exerted modest activities with an objective response rate of 16.7% and disease control rate of 46.3%, respectively [34]. In another trial, Janmmat et al. reported that gefitinib had demonstrated efficacy in patients with EGFR overexpression and ESCC histology as the second-line treatment [35]. Consistent with a previous report by Junk et al. [36], our studies demonstrated that ILQ had significantly inhibitory effects on the EGFR signaling pathway in esophageal squamous cell carcinoma. With the inactivation of EGFR, two key downstream molecules, ERK and Akt, were inhibited. In ILQ-treated tumor tissue, the phosphorylation of EGFR was substantially decreased. Moreover, in EGFR deficient cells, the sensitivities to ILQ were reduced significantly. All these results demonstrated that EGFR had important roles in ESCC development and is a crucial target for ILQ to exert its biological functions in ESCC.

In addition to the abnormality of EGFR activities, the dysregulation of the cell cycle is also important characteristic of ESCC. Cyclin D1 is a critical factor driving cell transition from G0 to G1 phase. By binding with cyclin-dependent kinase 4/6 (CDK4/6), cyclin D1 activates CDK4/6 and subsequently phosphorylates Rb, leading to the inactivation of Rb, which loses its function as cell cycle checkpoint [37]. Genomic profiling showed that CCND1 amplification was present in 57% tumor tissue and often coordinated with EGFR amplification to accelerate tumor progression [38, 39]. Some studies also indicated that dysregulated cyclin D1 expression is the reason for the reduced efficacy of EGFR inhibitors [40]. Therefore, we think that inhibiting EGFR activation and blocking cell cycle in ESCC simultaneously will take some advantages. Indeed, Zhou et al. showed that in ESCC the combination of CDK4/6 inhibitor and EGFR inhibitor had a significant synergistic effect and could prevent the resistance [41]. Excluding the inhibition of EGFR activity, through mediating the transcriptional activity of AP-1, ILQ also exerted significantly inhibitory effect on cyclin D1 expression. With the decrease of cyclin D1, ESCC cells were induced G0/G1 arrest after ILQ treatment. AP-1 is an essential transcriptional factor involved in the regulation of cyclin D1 expression [42]. In this study, the results of reporter gene assay demonstrated that the transcriptional activity of AP-1 was inhibited by ILQ. Western blotting also confirmed that the expression of proteins in Jun and Fos family was decreased after ILQ treatment. So we thought ILQ-mediated inhibition of AP-1 partially explained the mechanisms by which cyclin D1 was downregulated. On the other hand, because the regulation of AP-1 activity is complex and cyclin D1 expression was mediated due to different cellular contexts, therefore, more detailed investigations are needed to clarify the underlying mechanisms.

In summary, to the best of our knowledge, our studies for the first time investigated the antitumor activity of ILQ in ESCC. By suppression of EGFR signaling pathway and downregulated cyclin D1 expression, ILQ showed profound antitumor activities in ESCC. Our studies provided new insights into the role of ILQ in ESCC and the preclinical evidence for the clinical application of ILQ or its analogue.

## Figures and Tables

**Figure 1:** Isoliquiritigenin (ILQ) inhibited ESCC proliferation in vitro. (a) The structure of ILQ, B–D, ILQ inhibited ESCC cell proliferation. KYSE-140 (b), KYSE-520 (c), and TE-1 (d) cells were incubated with different concentrations of ILQ for different times, and cell viability was examined by MTS assay. E–G, ILQ inhibited the anchorage-independent growth of ESCC cells. KYSE-140 (e), KYSE-520 (f), and TE-1 (g) cells were treated with different ILQ, and the colony formation in soft agar was detected as described.

**Figure 2:** Isoliquiritigenin (ILQ) suppressed EGFR activation in ESCC cells. A ILQ inhibited EGFR signaling pathway. ESCC cells were treated with different ILQ for 2 h, and the expression of the indicated protein was detected by western blotting. B-C, ILQ blocked EGF-induced EGFR activation dose B and time C dependently. After starvation overnight, ESCC cells were incubated with ILQ for 2 h and then stimulated with 50 ng/ml EGF, the cell lysates were collected, and the expression of indicated protein was analyzed by western blotting. D–F, EGFR knockdown in ESCC cells impaired the sensitivity to ILQ, the expression of EGFR was silenced with shRNA(D) and then treated with ILQ.

**Figure 3:** Isoliquiritigenin (ILQ) decreased the transcriptional activity of AP-1. A-B, ILQ inhibited the expression of AP-1. KYSE-140 and TE-1 cells were treated with 10 *μ*M ILQ, and the expression of the indicated protein was examined by western blotting. C-D, ILQ decreased the transcriptional activity of AP-1. The pGL3-AP-1 vector was transfected into KYSE-140 or TE-1 cell and then treated with ILQ for 24 h; the transcriptional activity of AP-1 was detected as described. E, EGFR knockdown attenuated the inhibitory effect of ILQ on AP-1. KYSE-140 cells were infected with EGFR-shRNA and then transfected with pGL3-AP-1 vector; after the treatment of ILQ, the transcriptional activity of AP-1 was determined as described.

**Figure 4:** Isoliquiritigenin (ILQ) induced cell cycle arrested at the G0/G1 phase. (a) ILQ blocked the division of ESCC cells. KYSE-140 cell was treated with different ILQ for 24 h, and the expression of phosphor-histone H3 was detected by immunofluorescence. (b) ILQ induced G0/G1 cycle arrest. After treatment with ILQ for 24 h, the cells were stained with PI, and cell phased distribution was analyzed by FACS. (c) ILQ decreased the expression of cyclin D1. After the treatment of ILQ, the expression of indicated proteins was determined by western blotting.

**Figure 5:** Isoliquiritigenin (ILQ) inhibited tumor growth of xenograft in vivo. The KYSE-140 xenograft was established in nude mice and then treated with 10 mg/kg ILQ every two days. The antitumor ability was investigated. (a) The photograph of tumors; (b) the growth curve of xenograft; (c) the weight of tumors; (d) the body weight of tumor-bearing mice during in vivo experiment. (e) ILQ decreased phosphor-EGFR and Ki67 in tumor tissue. The phosphorylation of EGFR and Ki67 in ILQ-treated tumor tissue was analyzed by immunohistochemistry staining as described. Left, the representative photography; right, the expression of indicated markers was quantified.

**Figure 6:** The proposed antitumor mechanisms of ILQ in ESCC cells. With the suppression of EGFR activation, the activities of ERK1/2 and AKT were inhibited, leading to the decrease of AP-1 transcriptional activity and the reduction of cyclin D1 expression, which contributed to the G0/G1 cell cycle arrest.

## Data Availability

The data used to support the findings of this study are included within the article.
